# Relationship between microRNA-27a and efficacy of neoadjuvant chemotherapy in gastric cancer and its mechanism in gastric cancer cell growth and metastasis

This article has been retracted.

**DOI:** 10.1042/BSR20181175

**Published:** 2019-05-21

**Authors:** Chunlei Xu, Hong Cheng, Na Li, Ning Zhou, Xushan Tang

**Affiliations:** 1 Department of Digestive Internal Medicine, The Affiliated Tumor Hospital of Xinjiang Medical University, Wunumuqi 830053, P.R. China; 2 Department of Laboratory, The Affiliated Tumor Hospital of Xinjiang Medical University, Wunumuqi 830053, P.R. China

**Keywords:** Cell growth, Efficacy, Gastric cancer, Metastasis, MicroRNA-27a, Neoadjuvant chemotherapy

## Abstract

**Objective:** The aim of the present study is to investigate the relationship between microRNA-27a (miR-27a) and the efficacy of neoadjuvant chemotherapy in gastric cancer (GC) and its mechanism in the growth and metastasis of GC cells.

**Methods:** The expression of miR-27a in serum of 74 GC patients received neoadjuvant chemotherapy was detected by quantitative reverse transcriptase polymerase chain reaction (qRT-PCR). Clinical value and prognosis of miR-27a expression in predicting the efficacy of neoadjuvant chemotherapy in GC were evaluated. Besides, GC cells with low miR-27a expression were transfected with miR-27a mimics, and cells with high miR-27a expression were transfected with miR-27a inhibitors and secreted frizzled-related protein 1 (SFRP1) siRNA. A series of experiments were applied for the determination of cell viability, invasion and migration of GC cells.

**Results:** After neoadjuvant chemotherapy, the expression of miR-27a in serum of GC patients decreased significantly. Additionally, the expression of miR-27a in GC cell line was significantly higher than that in normal gastric mucosa cell line. Meanwhile, after down-regulating the expression of miR-27a in GC cells, the mRNA and protein expression of SFRP1 increased, the proliferation rate of cells slowed down, and the ability of invasion and migration decreased. Furthermore, combined with low expression of miR-27a and SFRP1, the proliferation rate of GC cells increased and the ability of invasion and migration increased.

**Conclusion:** Collectively, our study highlights that the high expression of miR-27a indicates the poor efficacy and prognosis of neoadjuvant chemotherapy in GC patients. Down-regulation of miR-27a can inhibit the growth and metastasis of GC cells via up-regulation of SFRP1.

## Introduction

Gastric cancer (GC) is known as one of the most frequent malignant tumors and ranks as the second leading cause of cancer-related mortalities around the world, especially in Asian countries [1,2]. As for the incidence of GC, there shows significant regional differences, and areas of the northwest and eastern coastal areas presenting with the highest incidence [3]. GC are both multi-step and multi-factor processes, and the development of which results from the combination of both genetic and epigenetic changes [4–6]. Early diagnosis is difficult for GC since it is often asymptomatic or it is manifested only moderate non-specific symptoms at the early stage, thus most patients will be at the advanced stages of GC upon first diagnosis [7–9]. Although surgery is considered as the mainstay of curative treatment, more than 50% patients with locally advanced GC recur even after complete resection [10]. Accordingly, investigators have demonstrated that neoadjuvant chemotherapy has been widely used in the treatment of advanced GC [11]. However, the effectiveness of neoadjuvant chemotherapy in patients with GC remains unpredictable. Therefore, novel biomarker detection is of significance for clinical practice of GC.

In recent years, convincing evidence has indicated that microRNAs (miRNAs) regulate many cellular processes associated with the biological behavior of tumors, such as cell proliferation, differentiation, metastasis and apoptosis [12,13]. It has also been suggested that miRNAs are involved in the progression of various malignant disease, including GC [14,15]. miRNAs, such as miR-214, miR-451, miR-130a and miR-27a have been regarded to be related to chemotherapy resistance [16–18]. Among which, miR-27a is located at chromosome 19, and the aberrant expressed miR-27a plays functional roles in many tumor types, such as esophageal cancer and renal cell carcinoma [19,20]. A previous study identifies a role for miR-27a in cell viability, invasion, migration and apoptosis through the activation of SFRP1-mediated Wnt/beta-catenin signaling in glioma [21]. Secreted frizzled-related protein (SFRPs), known as a tumor suppressor protein, is suggested to be a regulator of Wnt signaling pathway [22]. It has been reported that the overexpression of miR-27a in GC tissues and cells induces cell proliferation, migration as well as invasion via the activation of Wnt/β-catenin signaling pathway by binding to SFRP1 [23]. In view of the aforementioned results, we could speculate that the expression of miR-27a has correlation to the efficacy and prognosis of neoadjuvant chemotherapy in GC patients. Besides, down-regulation of miR-27a might inhibit the growth and metastasis of GC cells via up-regulation of SFRP1.

## Materials and methods

### Ethical statement

The present study was approved by the Human Research Ethics Committee of The Affiliated Tumor Hospital of Xinjiang Medical University, and written informed consent was obtained from all the subjects involved in the present study. In addition, the study was carried out in accordance with the World Medical Association Declaration of Helsinki.

### Study subjects

From March 2011 to March 2015, 74 patients with advanced GC (46 males and 28 females, with an average age of 58.7 ± 9.5 years) who had underwent neoadjuvant chemotherapy in The Affiliated Tumor Hospital of Xinjiang Medical University were enrolled into our experiment. The patients were included if they met the following criteria: 1. Patients were diagnosed with GC according to gastroscopy or cytology before operation. 2. According to the criteria for TNM staging at the seventh edition of International Union Against Cancer/American Joint Committee on Cancer (UICC/AJCC) in 2010, GC patients were classified into the advanced IIIB stage and IIIC stage. 3. Patients had not received any radiotherapy, chemotherapy or other adjuvant treatment prior to admission. 4. Patients had no chemotherapy contraindication. 5. According to the standards of the Response Evaluation Criteria in Solid Tumors (RECIST; 1.1) [24], patients had measurable lesions. Correspondingly, patients with distant metastasis, other malignant tumors, severe heart disease, arrhythmia or a history of myocardial infarction within a year or patients were pregnant or lactating women were excluded from our experiment.

### Neoadjuvant chemotherapy regimen and its efficacy evaluation

On the first day, patients were intravenously injected with 5% glucose solution containing 130 mg/m^2^ oxaliplatin, and from 1 to 14 days, 1000 mg/m^2^ capecitabine was given orally. A cycle for chemotherapy lasted for 21 days, with totally 3 cycles. Neoadjuvant chemotherapy was evaluated and re-operated after treatment. During intravenous chemotherapy, patients were treated with antiemetic drugs, while during oral chemotherapy, patients were given oral liver protection, Baiyao and neurotrophic drugs.

The evaluation of the efficacy of neoadjuvant chemotherapy was based on the criteria of RECIST 1.1: complete response (CR, all tumor lesions disappeared and lasted for 4 weeks); partial response (PR, the sum of the longest diameter of the tumor reduced more than 30% and lasts for 4 weeks); stable disease (SD, positioned between PR and PD); progressive disease (PD, the sum of the longest diameter of the tumor increased by 20%, or a new lesion appeared). The effective rate of chemotherapy was calculated as (CR + PR)/ total number of cases × 100%.

The venous blood samples were collected from patients before and after neoadjuvant chemotherapy, and the level of miR-27a in serum before and after neoadjuvant chemotherapy were detected by quantitative reverse transcriptase polymerase chain reaction (qRT-PCR).

#### Follow up

Patients were followed up by telephone, outpatient and medical records. The deadline of follow-up was March 2018, and five cases were lost to follow up from 3 to 36 months, and the follow-up rate was 93.2%. Progressive free survival (PFS) was defined as from the beginning time of treatment to the time of cancer recurrence or death.

### Cell selection and culture

GC cell lines (BGC-823, AGS, HGC-27, NCI-N87, SGC-7901, MKN45 and MGC-803) were purchased from Cell Resource Center of Shanghai Institutes for Biological Sciences of Chinese Academy of Sciences (China). Human normal gastric mucosal cell line GES-1 was purchased from Shanghai Aiyan Biotechnology Co., Ltd. (Shanghai, China). All the cells were cultured in a medium containing 10% fetal bovine serum (FBS) and 1% streptomycin (Gibco, Grand Island, NY, USA) at an incubator at 37°C with 5% CO_2_ as required. When the cell density reached about 80%, digestion and passage began. The expression of miR-27a in all cells was detected by qRT-PCR, and the appropriate cells were selected for follow-up experiment.

### Cell grouping and treatment

The GC cells (BGC-823 and MKN45) in logarithmic growth phase were treated with overexpression plasmids, and then assigned into groups: blank group, mimics negative control (NC) group (cells transfected with mimics NC), miR-27a mimics group (cells transfected with miR-27a mimics). Besides, the GC cells (SGC-7901 and AGS) in logarithmic growth phase were treated with poor expression plasmids, and then assigned into groups: blank group, inhibitors NC group (cells transfected with inhibitors NC), miR-27a inhibitors group (cells transfected with miR-27a inhibitors), miR-27a inhibitors + siRNA-NC group (cells transfected with miR-27a inhibitors and siRNA-NC) and miR-27a inhibitors + SFRP1-siRNA group (cells transfected with miR-27a inhibitors and SFRP1-siRNA). The mimics NC, miR-27a mimics, inhibitors NC, miR-27a inhibitors, siRNA-NC and SFRP1-siRNA were all purchased from Shanghai Gene Pharma Co., Ltd. (Shanghai, China). The cells were transfected according to the instructions of Lipofectamine 2000 (Invitrogen, Carlsbad, CA, USA). The cells were cultured in incubator for 48 h for further use.

### qRT-PCR

The total RNA in serum and cells was extracted by Trizol (Invitrogen, Carlsbad, CA, USA), and the high-quality RNA was confirmed by ultraviolet (UV) analysis and formaldehyde denaturation electrophoresis. cDNA was obtained by reverse transcription of avian myeloblastosis virus (AMV) reverse transcriptase from 1 μg RNA. PCR primers were designed and synthesized by Invitrogen Company (Carlsbad, CA, USA) (see Table 1) with glyceraldehyde phosphate dehydrogenase (GAPDH) or U6 as internal controls. The PCR amplification conditions were as follows: predenaturation at 94 °C for 5 min, with 40 cycles of denaturation at 94 °C for 40 s, annealing at 60 °C for 1 min and extension at 72 °C for 10 min. The product was verified by agarose gel electrophoresis. The threshold cycle (Ct) value of each reaction tube was obtained through the manual selection of the lowest point of parallel rise of each logarithmic expansion curve. The data were analyzed by 2^−ΔΔCt^ method, which was used for analyzing the ratio relation of target gene expression between the experimental group and the control group. ΔΔCt = [Ct_(target gene)_ − Ct_(internal control gene)_]_the experimental group_ − [Ct_(target gene)_ − Ct_(internal control gene)_]_the control group_. The experiment was repeated in triplicates.

**Table 1:** Primer sequence

Gene	Sequence
miR-27a	F: 5′-TTCACAGTGGCTAAG-3′
	R: 5′-GTGCAGGGTCCGAGGT-3′
U6	F: 5′- CTCGCTTCGGCAGCACA-3′
	R: 5′-AACGCTTCACGAATTTGCGT-3′
SFRP1	F: 5′-CGAGTTTGCACTGAGGATGA-3′
	R: 5′-CAGCACAAGCTTCTTCAGGTC-3′
GAPDH	F:5′-TGGGTGTGAACCATGAGAAG-3′
	R: 5′-GTGTCGCTGTTGAAGTCAGA-3′

Note: F, forward; GAPDH, glyceraldehyde phosphate dehydrogenase; miR-27a, microRNA-27a; R, reverse; SFRP1, secreted frizzled related protein 1.

### Western blot analysis

The proteins were extracted and the protein concentrations were determined referring to the instructions of the bicinchoninic acid (BCA) assay (Wuhan Boster Biological Technology LT, Wuhan, China). Next, the extracted protein was supplemented to the sample buffer and then boiled for 10 min at 95 °C (30 μg protein in each well). The protein samples were transferred to a nitrocellulose (NC) membrane using the wet transfer method following 10% sodium dodecyl sulfate polyacrylamide gel electrophoresis (SDS-PAGE) (Wuhan Boster Biological Technology LT, Wuhan, China), with the electrophoretic voltage from 80 V to 120 V, the transmembrane voltage of 100 mV as well as the time for 45–70 min. Afterwards, the protein samples were transferred to a polyvinylidene fluoride (PVDF) membrane and blocked with 5% bovine serum albumin (BSA). Subsequently, the membranes were added with the primary antibodies of SFRP1 (1:1000; Abcam, Cambridge, MA, USA) and β-actin (1:3000; Abcam, Cambridge, MA, USA) and then incubated at 4°C overnight. The membranes were rinsed with Tris-buffered saline and Tween 20 (TBST) three times, 5 min each, and then, the corresponding secondary antibodies (Shanghai Miao Tong Biotechnology Company, Shanghai, China) were incubated for 1 h at room temperature in order to wash the membranes three times, 5 min each. β-actin was regarded as an internal control. An electrogenerated chemiluminescence (ECL) solution together with Bio-rad Gel Dol EZ formatter (GEL DOC EZ IMAGER, Bio-rad, California, USA) was used for developing. The gray value of target band was analyzed by Image J software (National Institutes of Health, Bethesda, Maryland, USA). The experiment was repeated in triplicates.

### Cell counting kit-8 (CCK-8) assay

With a certain concentration, the cell suspensions of each group were diluted and then inoculated into 96-well plates at the density of 1 × 10^3^/100 μl/per well. Each group was set three multiple wells, and the culture plate was cultured at 37°C and 5% CO_2_. At the time point of 0 h, 24 h, 48 h, 72 h and 96 h, 10 μl cell counting kit-8 (CCK-8) solution was added to the corresponding well; and 10 μl CCK-8 solution was added to the cell-free medium as a blank control and incubated in an incubator for 4 h. The optical density of each well was measured at the wavelength of 450 nm. The experiment was repeated in triplicates.

### Transwell assay

The cells of each group were detached after 48-h transfection, *t*, and each Transwell chamber was spread in the ratio of 1: 8 Matrigel (80 μl) and seeded with 1 × 10^5^ cells. Next, the cells were added with 100 μl serum-free DMEM medium and the complete culture medium was added into the basolateral chamber and incubated for 24 h. After that, the cells in the apical chamber were erased with cotton swabs, fixed with 4% paraformaldehyde for 15 min, and stained with crystal violet for 10 min. Afterwards, five visual fields were selected for photographing and counting under a microscope. The number of invasive cells was the cells attached to the ventral side of the basement membrane. The experiment was repeated in triplicates.

### Scratch test

At the back of the six-well plate, a uniform horizontal line was drawn by a marker pen against the ruler about every 0.8 cm or so, crossing the well. Each well passed through at least five lines. When about 5 × 10^5^ cells were added into each well, the cell fusion rate reached 100%. On the next day, a 10 μl gun head was perpendicular to the back of the horizontal line against the ruler scratch. The gun head was vertical, which could not be tilted. The cells were gently washed with PBS three times after scratching, then gently adhered to the wall and added with PBS. The stretched cells were washed and removed, and then added to the culture medium and cultured in an incubator with CO_2_ at 37°C. The sampling was performed at the time point of 0 h and 24 h so as to take pictures under an inverted microscope. The wound healing area was calculated with National instrument Vision Assistant 8.6 software. Cell migration rate was calculated as the wound healing area/initial scratch wound area × 100. The experiment was repeated in triplicates.

### Double luciferase report gene assay

Bioinformatics software (http://www.targetscan.org) was used to predict the targeting relationship between miR-27a and SFRP1 and the binding sites between miR-27a and SFRP1 3′UTR. The sequence of SFRP1 3′UTR promoter containing miR-27a binding site was synthesized, and the SFRP1 3′UTR wild-type (WT) plasmid was constructed. On the basis of this plasmid, the SFRP1 3′UTR mutant (MUT) plasmid was constructed at the mutation binding site. According to the methods of the plasmid extraction kit (Promega, Madison, Wisconsin USA), the cells in the logarithmic growth were inoculated into 96-well plates and transfected with Lipofectamine 2000 at the cell density of about 70%. The plasmids of SFRP1-3′UTR-WT and SFRP1-3′UTR-MUT were mixed with mimics NC and miR-27a mimics (Shanghai GenePharma Co., Ltd, Shanghai, China), respectively, and then co-transfected into 293T cells. The cells were collected and lysed after 48 h of transfection. The luciferase activity was detected by luciferase detection kit (BioVision, San Francisco, CA, USA).

### Statistical analysis

SPSS 21.0 (SPSS, Inc, Chicago, IL, USA) software was applied for the analysis of all the data in our study. The Kolmogorov–Smirnov test verified the normal distribution of data. The results were expressed as mean ± standard deviation. The comparison between the two groups was analyzed by the *t* test, and the comparison among multiple groups was analyzed by the one-way analysis of variance (ANOVA). The Fisher’s least significant difference *t* test (LSD-*t*) was used for pairwise comparison. The clinical value of expression of miR-27a in neoadjuvant chemotherapy was evaluated by receiver operating characteristic (ROC) curve. Kaplan–Meier method and Log-rank test were used to analyze the relationship between the expression of miR-27a and the prognosis of neoadjuvant chemotherapy in patients with GC. All tests were two-sided and *P* values ≤ 0.05 were considered statistically significant.

## Results

### Decrease in miR-27a expression in serum of GC patients after neoadjuvant chemotherapy

The results of qRT-PCR showed that after three cycles of neoadjuvant chemotherapy, the expression of miR-27a in serum of GC patients decreased significantly (*P* < 0.05; Figure 1A), which suggested that the expression of miR-27a was related to neoadjuvant chemotherapy of GC.

**Figure 1:** Expression of miR-27a in serum of GC patients (**A**) Detection of miR-27a expression in serum of GC patients before and after neoadjuvant chemotherapy by qRT-PCR; (**B**) comparison of miR-27a expression in serum between the effective group and the ineffective group before neoadjuvant chemotherapy; *N* = 74; the *t* test was used for data analysis.

Among 74 GC patients after neoadjuvant chemotherapy, there were 3 cases in CR, 35 cases in PR, 24 cases in SD and 12 cases in PD. The effective rate of chemotherapy was 51.4%, that is, 38 patients were in the effective group and 36 in the ineffective group. After statistical analysis, the expression of miR-27a in serum of GC patients in the effective group was significantly lower than that of patients in the ineffective group (*P* < 0.05; Figure 1B), suggesting that the expression of miR-27a was related to the efficacy of neoadjuvant chemotherapy for GC.

### Efficiency analysis and prognostic significance of miR-27a expression in the prediction of neoadjuvant chemotherapy for GC

The area under curve (AUC) area of miR-27a expression in serum for predicting the efficacy of neoadjuvant chemotherapy of GC was 0.839, and the sensitivity and specificity was 72.2% and 89.5%, respectively (Figure 2A), which indicated that miR-27a expression had a good predictive effect on neoadjuvant chemotherapy efficacy in GC patients.

**Figure 2:** Relationship between miR-27a expression and the efficacy and prognosis of patients with GC after neoadjuvant chemotherapy (**A**) Diagnostic efficacy of serum miR-27a expression in patients with GC after neoadjuvant chemotherapy by ROC curve analysis; (**B**) expression of miR-27a in serum and prognosis of GC after neoadjuvant chemotherapy.

In order to analyze the relationship between the expression of miR-27a and the therapeutic effect of neoadjuvant chemotherapy in GC, the patients were divided into the high expression group (39 cases) and the low expression group (35 cases). After 36 months of follow-up, the median survival time of the high expression group was significantly lower than that of the low expression group (27.5 vs. 34.4; *P* < 0.05), which indicated that the expression of miR-27a was related to the efficacy of neoadjuvant chemotherapy in GC, and the prognosis of the low expression group was better after neoadjuvant chemotherapy (Figure 2B).

### High expression of miR-27a in GC cells

The results of qRT-PCR revealed that the expression of miR-27a in GC cell lines (BGC-823, AGS, HGC-27, NCI-N87, SGC-7901, MKN45 and MGC-803) was significantly higher than that in normal gastric mucosa cell line GES-1 (all *P* < 0.05; Figure 3A).

**Figure 3:** The difference of miR-27a expression between normal gastric mucosal cells and GC cells and the expression of miR-27a in GC cells after interfering with the expression of miR-27a (**A**) qRT-PCR was used to detect the expression of miR-27a in GC cells and normal gastric mucosal cells; (**B**) detection of transfection efficiency of miR-27a mimics in BGC-823 and MKN45 cells by qRT-PCR; (**C**) detection of transfection efficiency of miR-27a inhibitors in SGC-7901 and AGS by qRT-PCR; the experiment was repeated in triplicates; the comparison among multiple groups was analyzed by one-way ANOVA; the Fisher’s LSD-*t* was used for pairwise comparison; *, *P* < 0.05 compared with normal gastric mucosa cell or the blank group.

The expression of miR-27a in BGC-823 and MKN45 cells was lower among all the GC cell lines, so BGC-823 and MKN45 cells were selected to transfect miR-27a mimics. Compared with the blank group and the mimics NC group, the expression of miR-27a in the miR-27a mimics group was significantly increased (both *P* < 0.05; Figure 3B), which indicated that miR-27a mimics was transfected successfully.

The expression of miR-27a was higher in SGC-790 and AGS cells, and therefore, SGC-7901 and AGS cells were selected for miR-27a inhibitors transfection. In contrast with the blank group and the inhibitors NC group, the expression of miR-27a in the miR-27a inhibitors group was significantly decreased (both *P* < 0.05; Figure 3C), which indicated that miR-27a inhibitors was transfected successfully.

### Overexpression of miR-27a promotes proliferation, invasion and migration of GC cells

The results of MTT assay showed that in BGC-823 and MKN45 cells, there was no significant difference in cell proliferation between the blank group and the mimics NC group (*P* > 0.05), but the proliferation rate of GC cells in the miR-27a mimics group was higher than that of the blank group and the mimics NC group (both *P* < 0.05; Figure 4A,B).

**Figure 4:** Effects of overexpression of miR-27a on proliferation, invasion and migration of in BGC-823 and MKN45 cells (**A,B**) Detection of GC cell proliferation in BGC-823 and MKN45 cells by MTT assay; (**C,D**) Transwell assay was used to detect the invasion of BGC-823 and MKN45 cells (×200); (**E,F**) detection of migration of BGC-823 and MKN45 cells by scratch test; the experiment was repeated in triplicates; the comparison among multiple groups was analyzed by one-way ANOVA; the Fisher’s LSD-*t* was used for pairwise comparison; *, *P* < 0.05 compared with the blank group.

According to the results of Transwell assay, it was found that in BGC-823 and MKN45 cells, compared with the blank and mimics NC groups, the number of cell invasion of GC cells in the miR-27a mimics group was significantly increased (both *P* < 0.05; Figure 4C,D).

The results of scratch test showed that the cell migration rate of in BGC-823 and MKN45 cells in the miR-27a mimics group increased significantly in comparison with the blank group and the mimics NC group (both *P* < 0.05; Figure 4E,F).

### Low expression of miR-27a decreases proliferative, invasive and migratory potentials of GC cells

As shown in Figure 5A,B, MTT assay results showed that in SGC-7901 and AGS cells, there was no significant difference in cell proliferation of GC cells between the blank group and the inhibitors NC group (*P* > 0.05), but the proliferation rate of GC cells in the miR-27a inhibitors group was lower than that of the blank group and the inhibitors NC group (both *P* < 0.05).

**Figure 5:** Effects of decreased expression of miR-27a on proliferation, invasion and migration of SGC-7901 and AGS cells (**A,B**) Detection of GC cell proliferation of SGC-7901 and AGS cells by MTT assay; (**C,D**) Transwell assay was used to detect the invasion of SGC-7901 and AGS cells (×200); (**E,F**) detection of migration of SGC-7901 and AGS cells by scratch test; the experiment was repeated in triplicates; the comparison among multiple groups was analyzed by one-way ANOVA; the Fisher’s LSD-*t* was used for pairwise comparison; *, *P* < 0.05 compared with the blank group.

The findings of Transwell assay suggested that the number of cell invasion of SGC-7901 and AGS cells in the miR-27a inhibitors group was significantly decreased compared with the blank and inhibitors NC groups (both *P* < 0.05). There was no significant difference in cell invasion of GC cells between the blank group and the inhibitors NC group (*P* > 0.05; Figure 5C,D).

According to the results of scratch test, it was showed that the cell migration rate of SGC-7901 and AGS cells in the miR-27a inhibitors group decreased significantly in comparison with the blank group and the inhibitors NC group (both *P* < 0.05; Figure 5E,F).

### SFRP1 is determined as a target gene ofmiR-27a in GC cells

According to the finding of qRT-PCR and Western blot analysis, we found that in contrast with the normal gastric mucosa cell line GES-1, the mRNA and protein expression of SFRP1 was significantly decreased in GC cell lines (BGC-823, AGS, HGC-27, NCI-N87, SGC-7901, MKN45 and MGC-803) (all *P* < 0.05; Figure 6A,B).

**Figure 6:** The difference of SFRP1 expression between normal gastric mucosa cells and gastric carcinoma cells and the analysis of the expression of SFRP1 and the targeting relationship between miR-27a and SFRP1 in GC cells after interfering with the expression of miR-27a (**A**) Detection of mRNA expression of SFRP1 in various cells by qRT-PCR; (**B**) detection of SFRP1 protein expression in various cells by Western blot analysis; (**C**) effect of miR-27a mimics on SFRP1 mRNA expression by qRT-PCR; (**D**) effect of miR-27a mimics on SFRP1 protein expression detected by Western blot analysis; (**E**) effect of miR-27a inhibitors on SFRP1 mRNA expression by qRT-PCR; (**F**) effect of miR-27a inhibitors on SFRP1 protein expression detected by western blot analysis; (**G**) online prediction software and luciferase activity determination to verify the targeting relationship between miR-27a and SFRP1; the experiment was repeated in triplicates; the comparison among two or multiple groups was analyzed by the *t* test or the one-way ANOVA; the Fisher’s LSD-*t* was used for pairwise comparison; *, *P* < 0.05 compared with GES-1 cells or the mimics NC group.

After transfection of miR-27a mimics, the expression of SFRP1 mRNA and protein in GC cells decreased significantly, while the expression of SFRP1 mRNA and protein increased significantly after transfection of miR-27a inhibitors (both *P* < 0.05; Figure 6C–F).

Bioinformatics software (http://www.targetscan.org) predicts the targeting relationship between miR-27a and SFRP1. The results of luciferase activity test showed the luciferase activity in the SFRP1-3′UTR-WT + miR-27a mimics group was significantly lower than that in the SFRP1-3′UTR-WT + NC group (*P* < 0.05). However, there was no significant difference in luciferase activity between the SFRP1-3′UTR-MUT + NC group and the SFRP1-3′UTR-MUT + miR-27a mimics group (*P* >0.05; Figure 6G).

### SFRP1-siRNA reverses the inhibition effect of miR-27a inhibitors on GC cell proliferation, invasion and migration

Based on the aforementioned results, we have confirmed that miR-27a could regulate the growth and metastasis of GC cells and that miR-27a could inhibit the expression of SFRP1 in GC cells. Therefore, we hypothesized that miR-27a could regulate the growth and metastasis of GC cells by inhibiting the expression of SFRP1. Because of the high expression of miR-27a in GC cells, we set up the miR-27a inhibitors + SFRP1-siRNA group and used the miR-27a inhibitors + siRNA-NC group as the control to observe the change of cell growth and metastasis ability of GC cells. As shown in Figure 7A,B, the findings of MTT assay suggested that compared with the miR-27a inhibitors + siRNA-NC group, the proliferation rate of GC cells in the miR-27a inhibitors + SFRP1-siRNA group was significantly faster (*P* < 0.05).

**Figure 7:** Effects of low expression of miR-27a and SFRP1 on proliferation, invasion and migration of SGC-7901 and AGS cells (**A-B**) Detection of cell proliferation of SGC-7901 and AGS cells by MTT assay; (**C-D**) Transwell assay was used to detect the invasion of SGC-7901 and AGS cells (×200); (**E-F**) detection of migration of SGC-7901 and AGS cells GC cells by scratch test; the experiment was repeated in triplicates; the comparison between two groups was analyzed by the *t* test; *, *P* < 0.05 compared with the miR-27a inhibitors + siRNA-NC group.

The results of Transwell assay showed that the invasion ability of GC cells in the miR-27a inhibitors + SFRP1-siRNA group was significantly higher than that of the miR-27a inhibitors + siRNA-NC group, and the number of invasive cells in the miR-27a inhibitors + SFRP1-siRNA group increased significantly (*P* < 0.05; Figure 7C,D).

The results of scratch test indicated that the cell migration of GC cells in the miR-27a inhibitors + SFRP1-siRNA group was significantly higher than that in the miR-27a inhibitors + siRNA-NC group (*P* < 0.05; Figure 7E,F).

## Discussion

MiR-27a is a member of the well-identified miRNAs in tumors, and its diverse function is mainly depended on the cancer types, which could play a role either in promoting cancer or in tumor suppression [25–27]. Here, in this present study, we explored the mechanism by which miR-27a influences the carcinogenesis of GC. It was concluded from our study that expression of miR-27a was associated with the efficacy and prognosis of neoadjuvant chemotherapy in GC patients. Except that, down-regulation of miR-27a played an inhibitory role in the growth and metastasis of GC cells via up-regulation of SFRP1.

One of the most important findings in this present study demonstrated that expression of miR-27a was related to the efficacy of neoadjuvant chemotherapy for GC, and decreased miR-27a expression had a good predictive and prognostic effect on neoadjuvant chemotherapy efficacy in GC patients. The expression of several miRNAs has been suggested to be related to GC prognosis and could also evaluate the clinical response in some patients for neoadjuvant chemotherapy [28]. In accordance with the results in our study, miR-let-7a, miR-145 and miR-185 expression was remarkably decreased in GC patients after neoadjuvant chemotherapy, which supported that these mentioned miRNAs could have a potential role in assessing the efficacy of GC patients after neoadjuvant chemotherapy [11,29].

Generally, miRNAs exert their functions via the suppression of specific target genes [30]. For the purpose of finding a novel target gene through which miR-27a performs its effects in GC, we conducted an approach by using public bioinformatics tools. In our study, the results indicated that SFRP1 was a target gene of miR-27a. identify miR-27a can promote osteoblast differentiation by repressing a new target, SFRP1 expression at the transcriptional level [31]. Additionally, A dual-luciferase reporter assay was conducted to examine the effect of miR-27a on SFRP1, and the results suggested that miR-27a negatively regulated the expression of SFRP1 mRNA [32]. All these mentioned above reveals the target relationship between FRP1 and miR-27a.

Our study also demonstrates that the expression of miR-27a was significantly higher in GC tissues and cells, and low expression of miR-27a decreases proliferative, invasive and migratory potentials of GC cells. MiR-27a is considered as a carcinogenesis to be widely expressed in many tumors [33–35]. Liu et al. have elucidated that miR-27a was highly expressed in human MGC-803 GC cells [14], which is in accordance with our study. Besides, it was also supported by a report that a high expression of miR-27a was found in GC tissues in contrast with their matched non-tumor adjacent tissues [36]. Taken together, we have further demonstrated that miR-27a may act as an oncogene to be associated with carcinogenesis in human GC. In accordance with the results in this present study, a report has elucidated that down-regulation of miR-27a might suppress proliferation, migration as well as invasion of GC cells through binding to SFRP1 [23]. Additionally, the mechanism of miR-27a in the promoted proliferation of laryngeal carcinoma cells lies in that the binding site of miR-27a and its target gene could have great effect on 3′UTR of the prohibition gene, and based on this, miR-27a owns the function of oncogenes [25]. Guo et al. also suggested that that expression of SFRP1 might be silenced by miR-27a and based on which the tumor cell proliferation might be restricted, thereby resulting in the induction of apoptosis and differentiation [31].

In summary, the findings in our study has demonstrated that miR-27a was highly expressed in GC tissues and cells, and down-regulation of miR-27a played an inhibitory role in the growth and metastasis of GC cells via up-regulation of SFRP1. However, the specific mechanism of miR-27a targets SFRP1 in GC remains a future topic that needs to be further elucidated.

## Abbreviations

ANOVA: one-way analysis of variance
CCK-8: cell counting kit-8
CR: complete response
GC: gastric cancer
miR-27a: microRNA-27a
PR: partial response
RECIST: Response Evaluation Criteria in Solid Tumors
ROC: receiver operating characteristic
SD: stable disease
SDS-PAGE: sodium dodecyl sulfate polyacrylamide gel electrophoresis
SFRP1: secreted frizzled-related protein 1
WT: wild type
